RETRACTED

# A Retrospective Cohort Study of the Association Between Calcium Serum Level and Hypertension in Older Adults

**DOI:** 10.7759/cureus.40492

**Published:** 2023-06-16

**Authors:** Zia Sabah, Ahmed S Al Zomia, Mosab Deajim, Abdulrahman Alshahrani, Abdullah H Alamri, Ali M Alqahtani, Lama A Lahiq, Nasser A Alwaqdi, Berin Raj

**Affiliations:** 1 Department of Cardiology, King Khalid University, Abha, SAU; 2 College of Medicine, King Khalid University, Abha, SAU; 3 Department of Public Health, Prince Faisal Bin Khalid Cardiac Center, Abha, SAU; 4 Department of Public Health, University of Sunderland, Sunderland, GBR

**Keywords:** saudi arabia, adults, hypertension, calcium, creatine kinase, cardiac

## Abstract

Introduction: One of the major global risk factors for cardiovascular morbidity and death is hypertension. Earlier research has been conducted on the connection between calcium consumption and blood pressure.

Objective: This study aims to investigate the association between calcium serum levels and hypertension in older hypertensive adults.

Methods: A retrospective cohort study of 121 of hypertension patients was conducted in Prince Faisal Bin Khalid Cardiac Center. The data of all patients were collected by records, including lab, pathology, and medical review, in order to determine the effects on patients, providers, and institutions. Statistical analyses were performed using SPSS Statistics version 26.0. A p-value of <0.05 was considered statistically significant.

Results: The study included 121 adult hypertensive patients with a mean of age 60.29 ± 13.92. The majority of included patients were male (81%). More than one-third of patients were obese (39.7%), about one-third (33.9%) were overweight, and 26.4% of patients were in normal weight. The majority of patients had co-morbidities (68.3%); about one-half of them had diabetes mellitus (52.1%). The calcium level mean was 5.07 ± 1.26. The creatine kinase (CK) (initial day) mean ± SD was 813.22 ± 1146.37 became 221.4 ± 330.67 on the last day. The CK-myocardial band (CK-MB) (initial day) was 65.43 ± 118.9 and became 24.38 ± 23.26 on the last day. Additionally, the troponin (initial day) mean was 23.49 ± 104.26 and became 1.65 ± 2.66 on the last day. The most common discharge medications were anti-platelets (95%), beta-blockers (78.5%), statins (70.2%), and proton-pump inhibitors (PPI) (64.5%). The hospital stay days ranged from 1 to 20 days with a mean of 4.83 ± 3.38. The ICU stay days ranged from 1 to 15 days with a mean of 3.57 ± 2.72. Most of the patients (90.9%) improved.

Conclusion: There is no significant correlation between calcium levels in hypertensive patients and the demographic characteristics of patients, home or current medications, ECHO findings, or procedures done. However, there is a significant correlation between the calcium level and CK level among patients with hypertension. Further investigations are required to verify the relationship between CK and calcium levels in hypertensive patients.

RETRACTED

## Introduction

One of the major global risk factors for cardiovascular morbidity and death is hypertension [1]. Therefore, lifestyle changes are a crucial method for preventing and treating hypertension. According to earlier research, several lifestyle choices, including lowering salt intake, losing weight, drinking alcohol in moderation, and increasing physical exercise, can lower blood pressure (BP) [2].

Several studies have been conducted on the connection between calcium consumption and BP [1-3]. In experiments on animals, dietary calcium was shown to affect BP. For example, compared to rats fed a standard calcium diet, normotensive rats fed a free-calcium diet considerably elevated their systolic BP (SBP) between 15 and 35 mmHg [4-6]. Contrarily, calcium-supplemented normotensive and hypertensive rats showed significantly reduced SBP readings [6,7].

Increasing calcium consumption has been proven to reduce BP in both hypertensive and normotensive patients. SBP and diastolic BP (DBP) in normotensive adults were reported to be considerably decreased by dietary calcium treatments, such as supplementation or food fortification [6]. In hypertensive and normotensive populations, systematic reviews of calcium supplementation randomized controlled trials have demonstrated a consistent reduction in BP, with a mean difference in SBP of 2.5 mmHg in hypertensive subjects and 1.4 mmHg in normotensive subjects [8,9]. Even a little drop in BP was thought to be linked to a 10% decrease in stroke mortality and a 7% reduction in ischemic heart disease mortality in people [10].

In those under the age of 35 (2.11 mmHg) and with calcium dosages equal to or greater than 1500 mg/day (2.79 mmHg), the impact of calcium supplementation on SBP was greater. Because these studies only included around 20% of the participants, the stronger influence on BP decrease seen in these situations seems to have been diminished in the overall revision [11]. Most included studies were also conducted in high-income nations, where the average dietary calcium consumption is often higher [12]. The present study sought to investigate the association between calcium serum levels and hypertension in a cohort of older adults.

## Materials and methods

A retrospective cohort study was conducted at Prince Faisal Bin Khalid Cardiac Center, Abha, for Six months. One hundred hypertension patients were included in the study. The data of all patients were collected by Records including lab, pathology, and medical Review in order to determine the effects on patients, providers, and institutions.

RETRACTED

Statistical analyses

Statistical analyses were performed using SPSS Statistics version 26.0 (IBM Corp. Released 2019. IBM SPSS Statistics for Windows, Version 26.0. Armonk, NY: IBM Corp.) Categorical variables were presented using descriptive statistics, including total numbers and percentages. Comparison between categorical variables was analyzed using an x2 test. Continuous variables were presented as means + standard deviation (SD) if data were found to be normally distributed, with significant differences between the normally distributed continuous variables analyzed using the student's t-test. When data were not normally distributed, it was presented as median = interquartile range (IQR), with significant differences between the skewed continuous variables analyzed using the Mann-Whitney U Test. Testing for normality was performed using the Kolmogorov-Smirnov test. A p-value of <0.05 was considered statistically significant.

Ethical consideration

Informed consent was obtained before taking any information. Approval was obtained by the local Institutional Review Board committee of King Khaled University (ECM#2023-2006). Data were anonymous for patient confidentiality and used for research purposes only. The collected data were kept safely in a password-protected cloud.

## Results

The study included 121 hypertensive patients with a mean of age 60.29 ± 13.92. The patients were classified into four categories according to their age; patients <50 represented 24.8%, patients between 51 and 60 years represent 30.6%, patients between 61 and 70 years represent 22.3%, and patients older than 70 years represent 22.3% of the subjects. The majority of included patients were male (81%), while 19% were female. More than one-third of patients were obese (39.7%), about one-third (33.9%) were overweight, and 26.4% of patients were in normal weight. Hospital stay days of the included patients ranged from 1 to 20 days with a mean of 4.83 ± 3.38. ICU stay days of the included patients ranged from 1 to 15 days with a mean of 3.57 ± 2.72 (Table 1).

**Table 1:** Demographic characteristics of included hypertensive patients SD: standard deviation, IQR: interquartile range (range between 25th-75th percentiles), BMI: body mass index, ICU: intensive care unit

	Description (n=121)
Age (Y)	
Range	32 - 100
Mean ± SD	60.29 ± 13.92
Median (IQR)	59 (51 - 68)
Age (Y)	
< 50	30 (24.8)
51-60	37 (30.6)
61-70	27 (22.3)
>70	27 (22.3)
Gender	
Male	98 (81)
Female	23 (19)
BMI	
Underweight	0 (0)
Normal weight	32 (26.4)
Overweight	41 (33.9)
Obese	48 (39.7)
Hospital stay (days)	
Range	1 - 20
Mean ± SD	4.83 ± 3.38
Median (IQR)	4 (3 - 5)
ICU stay (days)	
Range	0 - 15
Mean ± SD	3.57 ± 2.72
Median (IQR)	3 (2 - 4)

Table 2 shows that the majority of patients had co-morbidities (68.3%); about one-half of them had diabetes mellitus (52.1%). The most common medications of the included hypertensive patients were beta-blockers (83.5%), angiotensin-converting enzyme inhibitors (55.4%), and diuretics (43%). Most of the patients (90.9%) improved.

RETRACTED

**Table 2:** Clinical characteristics of included hypertensive patients ACE: angiotensin-converting enzyme, ARBs: angiotensin receptor blockers, PPI: proton-pump inhibitor, DM: diabetes mellitus, HTN: hypertension, CCB: calcium channel blocker

	Description (n=121)
Home medications	
Anti-platelets	15 (12.4)
Beta-blockers	8 (6.6)
ACE inhibitors	8 (6.6)
ARBs	8 (6.6)
Statin	18 (14.9)
Diuretics	6 (5)
Insulin	18 (14.9)
PPI	10 (8.3)
Presence of co-morbidity	83 (68.6)
DM	63 (52.1)
HTN	52 (43)
Current medications	
Diuretics	52 (43)
CCB	10 (8.3)
ARB	22 (18.2)
ACE inhibitors	67 (55.4)
Beta-blockers	101 (83.5)
Status	
The same	3 (2.5)
Improved/stable	118 (97.5)
Outcome	
The same	11 (9.1)
Improved/stable	110 (90.9)

Table 3 shows that the most common ECHO findings in the included hypertensive patients were valve affection (83.5%) and mitral reg (79.3%), followed by tricuspid regurgitation (TR) (39.7%) and ejection fraction (EF) <40% (33.1%). Percutaneous coronary intervention (PCI) was carried out on 58.7% of the included patients, and coronary artery bypass grafting (CABG) and coronary angiography (CAG) were carried out on 9.1% of patients. Balloon valvuloplasty (1.7%), percutaneous transluminal coronary angioplasty (PTCA) (4.1%), implantable cardioverter-defibrillator (ICD) insertion (3.3%), or medical treatment (8.3%) were also carried out on some patients. The most common discharge medications were anti-platelets (95%), beta-blockers (78.5%), statins (70.2%), and PPIs (64.5%).

**Table 3:** ECHO findings and procedure did to the hypertensive patients EF: ejection fraction, TR: tricuspid regurgitation, aortic st: aortic stenosis, aortic reg: aortic regurgitation, CABG: coronary artery bypass grafting, PCI: percutaneous coronary intervention, CAG: coronary angiography, PTCA: percutaneous transluminal coronary angioplasty, ICD: implantable cardioverter-defibrillator, ACE: angiotensin-converting enzyme, ARBs: angiotensin receptor blockers, PPI: proton-pump inhibitor

	Description (n=121)
ECHO findings	
EF <40%	40 (33.1)
Valve affection	101 (83.5)
Mitral Reg	96 (79.3)
TR	48 (39.7)
Aortic St	2 (1.7)
Aortic Reg	11 (9.1)
Procedure done	
CABG	11 (9.1)
PCI	71 (58.7)
CAG	11 (9.1)
Balloon valvuloplasty	2 (1.7)
PTCA	5 (4.1)
ICD insertion	4 (3.3)
Medical treatment	10 (8.3)
Discharge medication	
Anti-platelets	115 (95)
Beta-blockers	95 (78.5)
ACE inhibitors	57 (47.1)
ARBs	30 (24.8)
Statin	85 (70.2)
Diuretics	41 (33.9)
Insulin	4 (3.3)
PPI	78 (64.5)

Table 4 shows the laboratory tests that were carried out on the included hypertensive patients including hemoglobin (HB), platelets, hematocrit (HCT), kidney functions, calcium, electrolytes, creatine kinase (CK), CK-myocardial band (CK-MB), and troponin (TROP). The calcium level mean was 5.07 ± 1.26. The CK (initial day) mean ± SD was 813.22 ± 1146.37 and on the last day was 221.4 ± 330.67. The CK-MB (initial day) was 65.43 ± 118.9 and on the last day was 24.38 ± 23.26. Additionally, the TROP (initial day) mean was 23.49 ± 104.26 and on the last day was 1.65 ± 2.66.

RETRACTED

**Table 4:** Laboratory tests of the included hypertensive patients SD: standard deviation, IQR: interquartile range (range between 25th-75th percentiles), HCT: hematocrit, CK: creatine kinase, CK-MB: creatine kinase-myocardial band, TROP: troponin

	Description (n=121)
HB	
Range	8.36-18.73
Mean ± SD	14.5 ± 2.27
Median (IQR)	14.56 (13.09-16.02)
Platelets	
Range	14.5-905.8
Mean ± SD	280.99 ± 132.76
Median (IQR)	250 (201-336.2)
HCT	
Range	13.28-215.7
Mean ± SD	45.59 ± 18.39
Median (IQR)	44.06 (39.29-48.8)
Uric acid (init)	
Range	2.75-13.82
Mean ± SD	6.29 ± 2
Median (IQR)	6.16 (4.98-7.4)
Uric acid (X day)	
Range	2.7 - 14.81
Mean ± SD	6.6 ± 2.19
Median (IQR)	6.24 (5-7.58)
Uric acid (X day)	
Range	2.43-15.25
Mean ± SD	6.66 ± 2.34
Median (IQR)	6.28 (4.8-7.92)
Uric acid (X day) 2	
Range	2.78-16.13
Mean ± SD	6.96 ± 2.79
Median (IQR)	6.5 (4.88-8.12)
Uric acid (last)	
Range	2.55-17.17
Mean ± SD	6.55 ± 2.77
Median (IQR)	5.85 (4.8-7.56)
Calcium	
Range	2.07-12.39
Mean ± SD	5.07 ± 1.26
Median (IQR)	4.82 (4.7-4.94)
Phosph	
Range	0.5-5.97
Mean ± SD	3.27 ± 0.88
Median (IQR)	3.36 (2.77-3.7)
Sodium	
Range	2.41-158
Mean ± SD	134.54 ± 12.99
Median (IQR)	136 (133-138)
Potassium	
Range	2.29-5.16
Mean ± SD	4.13 ± 0.48
Median (IQR)	4.17 (3.88-4.46)
Urea	
Range	9.82-163.95
Mean ± SD	43.88 ± 27.76
Median (IQR)	37.1 (28.28-47.16)
Creatinine	
Range	0.44-3.1
Mean ± SD	1.12 ± 0.41
Median (IQR)	1.05 (0.88-1.21)
CK (initial)	
Range	29.2-4978.2
Mean ± SD	813.22 ± 1146.37
Median (IQR)	274.35 (91.45-1005.09)
CK (X day)	
Range	26-4008.6
Mean ± SD	529.72 ± 775.17
Median (IQR)	183.65 (90.45-740.8)
CK (X day)	
Range	20.72-2289.4
Mean ± SD	314.13 ± 432.55
Median (IQR)	155 (82.5-346.8)
CK (X day) 3	
Range	24.57-1685.79
Mean ± SD	234.92 ± 330.23
Median (IQR)	114.1 (62.8-279.9)
CK (last day)	
Range	19.48-1804.8
Mean ± SD	221.4 ± 330.67
Median (IQR)	97.78 (58.1-227)
CK-MB (initial)	
Range	4.45-1530.5
Mean ± SD	121.09 ± 198.13
Median (IQR)	35.34 (19.7-146.87)
CK-MB (X day)	
Range	2.14-866.35
Mean ± SD	65.43 ± 118.9
Median (IQR)	28.39 (16.62-62.69)
CK-MB (X day) 4	
Range	1.9-282.7
Mean ± SD	33.73 ± 35.08
Median (IQR)	25.03 (16.39-41.57)
CK-MB (X day)	
Range	5.76-73
Mean ± SD	25.56 ± 16.95
Median (IQR)	20.29 (13.57-30.74)
CK-MB (last day)	
Range	6.9-146.75
Mean ± SD	24.38 ± 23.26
Median (IQR)	18.71 (11.33-27)
TROP (initial)	
Range	0-725
Mean ± SD	23.49 ± 104.26
Median (IQR)	1.5 (0.05-12)
TROP (last day)	
Range	0-11.05
Mean ± SD	1.65 ± 2.66
Median (IQR)	0.78 (0.02-1.96)

Table 5 shows that there is no significant correlation (P>0.05) between the calcium level of the hypertensive patients and the demographic characters of patients, home or current medications, ECHO findings, or procedures done.

RETRACTED

**Table 5:** Correlation between calcium and other qualitative variables BMI: body mass index, ACE: angiotensin-converting enzyme, ARBs: angiotensin receptor blockers, PPI: proton-pump inhibitor, DM: diabetes mellitus, HTN: hypertension, CCB: calcium channel blocker, ARB: angiotensin receptor blocker, EF: ejection fraction, mitral reg: mitral regurgitation, TR: tricuspid regurgitation, aortic st: aortic stenosis, aortic reg: aortic regurgitation, CABG: coronary artery bypass grafting, PCI: percutaneous coronary intervention, CAG: coronary angiography, PTCA: percutaneous transluminal coronary angioplasty, ICD: implantable cardioverter-defibrillator

	Calcium	
	Mean ± SD	p-value
Age (Y)		
<50	4.7 ± 0.6	0.130
51-60	4.8 ± 0.9	
61-70	5.2 ± 1.2	
>70	5.7 ± 2	
Gender		
Male	5 ± 1.1	0.127
Female	5.4 ± 1.8	
BMI		
Normal weight	5 ± 1.1	0.413
Overweight	4.9 ± 1	
Obese	5.3 ± 1.6	
Home medications		
Anti-platelets		
Yes	4.8 ± 0.2	0.866
No	5.1 ± 1.4	
Beta-blockers		
Yes	5.4 ± 1.3	0.663
No	5 ± 1.3	
ACE inhibitors		
Yes	4.9 ± 0.2	0.557
No	5.1 ± 1.3	
ARBs		
Yes	4.9 ± 0.2	0.211
No	5.1 ± 1.3	
Statin		
Yes	5 ± 0.8	0.931
No	5.1 ± 1.3	
Diuretics		
Yes	5.5 ± 1.4	0.367
No	5 ± 1.3	
Insulin		
Yes	5 ± 0.9	0.488
No	5.1 ± 1.3	
PPI		
Yes	5.2 ± 1.1	0.638
No	5.1 ± 1.3	
Co-morbidity		
Yes	5.2 ± 1.4	0.669
No	4.7 ± 0.5	
DM		
Yes	5 ± 1.1	0.846
No	5.1 ± 1.5	
HTN		
Yes	5.3 ± 1.6	0.245
No	4.8 ± 0.9	
Current medications		
Diuretics		
Yes	5.1 ± 1.2	0.659
No	5 ± 1.3	
CCB		
Yes	5.6 ± 2.5	0.709
No	5 ± 1.1	
ARB		
Yes	5.4 ± 1.4	0.239
No	5 ± 1.2	
ACE inhibitor		
Yes	5 ± 1	0.150
No	5.1 ± 1.5	
Beta-blocker		
Yes	5 ± 1.1	0.209
No	5.3 ± 1.9	
Status		
The same	5.9 ± 2.1	0.849
Improved/stable	5 ± 1.2	
Outcome		
The same	5.2 ± 1.1	0.730
Improved/stable	5.1 ± 1.3	
ECHO findings		
EF		
<40%	4.9 ± 0.6	0.692
40% or more	5.1 ± 1.5	
Valve affection		
Yes	5.1 ± 1.3	0.476
No	4.9 ± 1.3	
Mitral Reg		
Yes	5.1 ± 1.3	0.281
No	5.1 ± 1.3	
TR		
Yes	5.5 ± 1.7	0.518
No	4.8 ± 0.8	
Aortic St		
Yes	4.8 ± .	0.680
No	5.1 ± 1.3	
Aortic Reg		
Yes	4.8 ± 1.3	0.431
No	5.1 ± 1.3	
Procedure done		
CABG		
Yes	5.5 ± 1.5	0.791
No	5 ± 1.2	
PCI		
Yes	4.9 ± 0.7	0.835
No	5.3 ± 1.7	
CAG		
Yes	4.5 ± 0.9	0.298
No	5.1 ± 1.3	
Balloon valvuloplasty		
Yes	4.9 ± .	0.800
No	5.1 ± 1.3	
PTCA		
Yes	4.7 ± 0.2	0.420
No	5.1 ± 1.3	
ICD insertion		
Yes	5.1 ± .	0.300
No	5.1 ± 1.3	
Medical treatment		
Yes	5.4 ± 1.4	0.664
No	5 ± 1.3	
Discharge medication		
Anti-platelets		
Yes	5 ± 1.2	0.278
No	5.8 ± 2.2	
Beta-blockers		
Yes	5 ± 1	0.771
No	5.3 ± 2	
ACE inhibitors		
Yes	4.9 ± 0.5	0.146
No	5.2 ± 1.6	
ARBs		
Yes	5.3 ± 1.6	0.394
No	5 ± 1.1	
Statin		
Yes	5.1 ± 1.4	0.921
No	4.9 ± 0.9	
Diuretics		
Yes	5.2 ± 1.3	0.385
No	5 ± 1.3	
Insulin		
Yes	4.8 ± 0.1	0.879
No	5.1 ± 1.3	
PPI		
Yes	5.2 ± 1.4	0.796
No	4.9 ± 0.9	

Table 6 shows that there is a significant correlation (P<0.05) between the calcium level and CK level among patients with hypertension.

RETRACTED

**Table 6:** Correlation between calcium and other quantitative variables r: Spearman correlation coefficient, P: p-value, ICE: intensive care unit, HB: hemoglobin, HCT: hematocrit, CK: creatine kinase, CK-MB: creatine kinase-myocardial band, TROP: troponin

	Calcium	
	r	p-value
Age (Y)	0.113	0.261
Hospital stay (days)	0.153	0.128
ICU stay (days)	0.079	0.470
HB	0.078	0.442
Platelets	0.048	0.632
HCT	0.156	0.122
Uric acid (init)	0.051	0.619
Uric acid (X day)	0.123	0.251
Uric acid (X day)	0.141	0.224
Uric acid (X day) 2	0.101	0.491
Uric acid (last)	0.107	0.411
Phosph	0.144	0.188
Sodium	-0.098	0.333
potassium	0.050	0.621
urea	0.080	0.433
Creatinine	0.028	0.782
CK (initial)	-0.185	0.072
CK (X day)	-0.240	0.031
CK (X day)	-0.283	0.018
CK (X day) 3	-0.397	0.018
CK (last day)	-0.331	0.013
CK-MB (initial)	-0.061	0.562
CK-MB (X day)	-0.122	0.276
CK-MB (X day) 4	-0.024	0.852
CK-MB (X day)	-0.025	0.882
CK-MB (last day)	0.090	0.510
TROP (initial)	-0.113	0.293
TROP (last day)	0.133	0.555

## Discussion

Over the past two decades, there has been a rise in the prevalence of hypertension worldwide [13]. According to specific research, dietary behaviors and the risk of developing hypertension have been associated [14,15]. According to several studies, the consumption of dairy products is inversely related to both BP levels and the risk of developing hypertension [16-18]. However, a long-term relationship between dietary calcium consumption and the risk of developing hypertension has not yet been proven. The current study aims to investigate the association between calcium serum levels and hypertension in older adults.

RETRACTED

The majority of included patients had co-morbidities (68.3%); about one-half of them had diabetes mellitus (52.1%). Diabetes mellitus and hypertension frequently coexist. Diabetes mellitus is a significant risk factor for cardiovascular diseases, increasing the risk in people with hypertension. Although hypertension and diabetes mellitus may be diagnosed simultaneously, many instances of hypertension occurring before the development of diabetes mellitus may indicate that it develops on its own or as a result of metabolic syndrome [19,20].

The most common medications of the included hypertensive patients were beta-blockers (83.5%), ACE inhibitors (55.4%), and diuretics (43%). Most of the patients improved. The most commonly used medications reported by hypertensive patients were angiotensin receptor antagonists, calcium channel blockers, ACE inhibitors, beta-blocker, alpha-blockers, thiazide, and non-thiazide diuretics [21,22].

According to the present results, the most common ECHO findings in the included hypertensive patients were valve affection (83.5%) and mitral reg (79.3%), TR (39.7%) and EF <40% (33.1%). PCI was performed on 58.7% of the included patients; CABG and CAG were performed on 9.1%. Balloon valvuloplasty (1.7%), PTCA (4.1%), ICD insertion (3.3%), or medical treatment (8.3%) were also carried out on some patients. The most common discharge medications were anti-platelets (95%), beta-blockers (78.5%), statins (70.2%), and PPIs (64.5%). The laboratory tests carried out on hypertensive patients included HB, platelets, HCT, kidney functions, calcium, electrolytes, CK, CK-MB, and TROP.

The present study demonstrated no significant correlations between calcium level in hypertensive patients and demographic characteristics of patients, home or current medications, ECHO findings, or procedures done; however, a significant correlation between the calcium level and CK level among patients with hypertension. One study by Lee et al. (2017) showed that a high coronary calcium score with post-procedural CK-MB might be a valuable predictor for TLR after DES implantation [22]. Previous research found that blood CK activity can significantly rise without any clinically evident cardiac or skeletal muscle disorders when there is hypocalcemia. Patients with hypocalcemia have significant individual variations in serum CK activity. In situations of severe hypocalcemia, high CK activity is more likely to occur [23-25].

Study Limitations

Several limitations to this study should be considered when interpreting the results. Firstly, the study is a retrospective cohort study, which relies on data collected from medical records rather than from a controlled experimental design. This can introduce potential biases and confounding variables that may affect the validity of the findings. Secondly, the study only included a relatively small sample size of 121 hypertensive patients from a single cardiac center, which may limit the generalizability of the findings to other populations. Thirdly, the study only measured serum calcium levels at a single time point and did not assess changes in calcium intake over time. This may limit the ability to establish a causal relationship between calcium intake and hypertension. Fourthly, the study did not control for other dietary factors affecting BP, such as sodium intake, which may have confounded the results. Lastly, the study did not investigate the potential mechanisms underlying the observed relationship between calcium and CK levels, which may be necessary for understanding the clinical implications of these findings.

RETRACTED

## Conclusions

The present study demonstrated no significant relationship between calcium level in hypertensive patients and demographic characteristics of patients, home or current medications, ECHO findings, or procedures done; however, a significant correlation between the calcium level and CK level was found among patients with hypertension. Previous research found that blood CK activity can significantly rise without any clinically evident cardiac or skeletal muscle disorders when there is hypocalcemia. However, it is unknown how serum CK activity is increased by hypocalcemia. Therefore, further investigations are required to study the relationship between CK and calcium levels in hypertensive patients.
